# A Novel Hadoop Security Model for Addressing Malicious Collusive Workers

**DOI:** 10.1155/2021/5753948

**Published:** 2021-07-08

**Authors:** Amr M. Sauber, Ahmed Awad, Amr F. Shawish, Passent M. El-Kafrawy

**Affiliations:** ^1^Faculty of Science, Menoufia University, Shibin Al Kawm, Egypt; ^2^University of Tartu, Tartu, Estonia; ^3^Cairo University, Giza, Egypt; ^4^School of Information Technology and Computer Science, Nile University, Giza, Egypt

## Abstract

With the daily increase of data production and collection, Hadoop is a platform for processing big data on a distributed system. A master node globally manages running jobs, whereas worker nodes process partitions of the data locally. Hadoop uses MapReduce as an effective computing model. However, Hadoop experiences a high level of security vulnerability over hybrid and public clouds. Specially, several workers can fake results without actually processing their portions of the data. Several redundancy-based approaches have been proposed to counteract this risk. A replication mechanism is used to duplicate all or some of the tasks over multiple workers (nodes). A drawback of such approaches is that they generate a high overhead over the cluster. Additionally, malicious workers can behave well for a long period of time and attack later. This paper presents a novel model to enhance the security of the cloud environment against untrusted workers. A new component called malicious workers' trap (MWT) is developed to run on the master node to detect malicious (noncollusive and collusive) workers as they convert and attack the system. An implementation to test the proposed model and to analyze the performance of the system shows that the proposed model can accurately detect malicious workers with minor processing overhead compared to vanilla MapReduce and Verifiable MapReduce (V-MR) model [1]. In addition, MWT maintains a balance between the security and usability of the Hadoop cluster.

## 1. Introduction

The distributed MapReduce (MR) model provides parallelism for large-scale data processing, a Google project introduced by Apache Hadoop [2]. It was developed by Doug Cutting and Mike Cafarella in 2005, an open-source implementation of a high-performance computing model. It is globally used by large-scale companies. For instance, Amazon implemented the Hadoop cluster with MapReduce as a public service available for research and/or data analytics on big data [3]. MR provides applications to work on thousands of machines and petabytes of information in parallel and in a cost-effective manner. This is accomplished by using commodity hardware to build cluster nodes as core basic components of Hadoop [4–7]. A Hadoop Cluster consists of a single master node that hosts the JobTracker service and a set of workers each hosting a TaskTracker service. There are two components of the Hadoop framework: MapReduce and HDFS. HDFS transfers an amount of data very rapidly to MapReduce and its components combine to support applications with large data sets as shown in Figure 1.

Accordingly, such systems face integrity issues since worker nodes can be on different, possibly untrusted domains [8]. Those public workers might be malicious or become malicious over time, sending wrong results as a main security threat to the whole system. The common approach to pick such behavior is redundantly outsourcing tasks on different workers in different domains and then comparing results [9].

For scalability, clusters can be composed of machines on private and/or public networks. Using machines in the public cloud hinders the security of the total system [10]. Thus, we need to test each node whether it can be trusted by validating that the node is not malicious. What makes it hard to detect malicious workers is the fact that they keep acting normally until they gain trust. Then, they turn malicious, on the one hand. On the other hand, malicious workers are detected by replication of given jobs and comparing the results. As a workaround from malicious workers, such workers can cooperate to consistently return wrong results, which makes malicious workers' detection very hard. Moreover, replication consumes more resources leading to higher costs and longer waiting times for other jobs. Malicious workers are the attackers classified into two categories based on their behavior, noncollusive and collusive workers [11]. They can cheat on a task by giving a wrong result or tamper with the intermediate outputs to mess up the final result. Noncollusive ones behave independently to destruct the work of the system, whereas collusive workers cooperate together to deceive the system until they are trusted and then attack. If trusted workers are known based on comparing the results returned, then collusive ones are hard to detect as the comparison of replicated tasks will be inconclusive with respect to worker trustworthiness.

Existing solutions for detecting harmful workers in public MR clouds are not sufficiently effective [12]. In recent years, many researchers have worked in this area to increase the security of systems and cloud computing. In order to ensure the accuracy of the computation, several frameworks have been designed, including SecureMR [12], VIAF [11], weighted t-first voting [13], IntegrityMR [14], Accountable MR [15], TS-TRV [16], and Verifiable MapReduce (V-MR) [1]. The goal is to detect malicious workers and mark them out to guarantee the integrity of the results. Those techniques suffer from high overhead costs due to repeated processing. Moreover, not all types of malicious workers can be detected.

This paper proposes a novel solution: the Malicious Worker Trap (MWT). It is both more effective and efficient compared to the state of the art. That is, it has a much lower processing overhead (efficiency) in detecting both collusive and noncollusive workers (effectiveness). MWT is an added service on the master node parallel to the NameNode and JobTracker, communicating with both of them. NameNode keeps the directory tree of all files in the file system and tracks data files across the cluster while the JobTracker schedules jobs submitted for execution. The new service shall send extra jobs to the JobTracker interleaving with the original ones to be assigned to workers for verification. In this paper, we present a new service on the master node of Hadoop MapReduce. The following are the main contributions of this paper:

- A lightweight malicious worker detection approach (MWT) that is capable of detecting both collusive and noncollusive malicious workers
- Implementation of MWT as a service within Hadoop's master node
- An evaluation of the approach with respect to processing overhead compared to Vanilla Hadoop and state-of-the-art V-MR model that uses work replication

## 2. Background and Related Work

To ensure the integrity of the MR computations, researchers developed a number of frameworks. They concentrated on improving the functionality of mappers and reducers in terms of security. As intruders try to hinder the computations of the mappers and reducers, they need to be elicited to ensure the correctness of the results. In open systems, common collude behavior can be summarized according to the following attacks [11, 12, 14, 15, 17]. A bad worker may

1. Cheat on a task by giving the wrong result without processing the input or may tamper the intermediate result to mess up the final result
2. Launch DoS attacks against other good workers. For example, it may keep sending requests to a good worker and ask for intermediate results or it may impersonate the master and send fake assignments to good workers
3. Initiate replay attacks against good workers by sending old task assignments to keep them busy
4. Eavesdrop and tamper the messages exchanged between the master node and the workers to invalidate the final results

The second and third attacks can be solved normally by common cloud security mechanisms [12, 18–20]. However, the first and the fourth are the ones that are hard to detect.

Detecting and preventing passive network eavesdropping attacks are extremely difficult, if not impossible, as there are no disruptions or changes to the network. Active attacks are easier to detect, but often, data is already intercepted by the time network changes are noticed. There are methods to overcome the exchanged Eavesdropped and tampered messages between the master node and the workers such as

1. Encryption: first and foremost, encrypt e-mail, networks, and communications, as well as data at rest between the master node and slave nodes, in use and in motion. That way, even if data is intercepted, the hacker will not be able to decrypt it without the encryption key.
2. Authentication: authenticating incoming packets is key to preventing spoofed packets that are used to perpetrate IP spoofing or MAC address spoofing attacks. Use standards and protocols that provide authentication for master node and DataNodes.
3. Network monitoring: security teams should constantly monitor networks for abnormal activity by using intrusion detection systems or endpoint detection and response software. Security teams use the same sniffer programs that nefarious actors use to detect vulnerabilities on the network.

Malicious workers can attack as independent workers or as a group of workers. Those are called noncollusive and collusive, respectively, as discussed in Section 1.

Detection approaches include grouping and weighing [13], replication-based detection [11], quiz and testing [11], voting [21], and multiple clouds [14].

### 2.1. Multiple Clouds' Technique

The cluster computing model of MR is expanded to span multiple public and or private clouds [22]. Based on such architecture, IntegrityMR [14] is an integrity assurance framework for analyzing big data and managing applications. The IntegrityMR solution covers the MR framework on a hybrid cloud (public and private clouds). This was the first method that provided multiple public cloud architectures for MR computing. In addition, it is the first method to ensure the correctness of the result without much change in MR's work. In task assignment, instead of picking a worker from the single public cloud, IntegrityMR can randomly choose a public cloud and pick a worker from the chosen cloud. Randomized task assignment would bear significant performance overhead due to the existence of the shuffle phase, where the mappers send their intermediate results to the reducer. It is likely that the mappers and the reducers are not in the same cloud. This means intercluster data transmission, possibly over the Internet. This will slow down the overall computation. They solve this problem by having the master assign the original map tasks and reduce tasks to the same cloud and the replicated map tasks and reduce tasks to another cloud. Since the reducer only accepts map results from the same cloud, shuffle would only happen inside a cloud. For this framework to be effective, a private cloud must be used as a verifier. Thus, this is an expensive solution.

In [14], the authors proposed a Cross-Cloud MapReduce (CCMR) framework that adds integrity checks in the mapper and reducer phases. In the map phase, an integrity check is performed on map tasks. In the reduce phase, CCMR factors each reduce task into multiple subtasks and apply the integrity check on the subtasks. To achieve high integrity, reduce tasks are executed on the private cloud to detect infringements. Again, this incurs high data transmission costs and the unavoidable dependency on private clouds for verification.

Yoon and Liu [1] presented a solution called Verifiable MapReduce (V-MR) that verifies the integrity of MapReduce computations via partial reexecutions. The approach is composed of two stages: online tracing and offline verification. Online tracing is to record execution traces of the user-defined MapReduce application on every worker node during normal execution. The offline verifier analyzes the execution traces to identify and select the requests to reexecute and prepare the new code and the input data for partial reexecution. Compared to the two previous approaches, it is more efficient as it does not require heavy data transfers and it can decide about integrity via partial results on carefully selected subsets of the data.

### 2.2. Quiz and Testing Technique

In this type of approaches, one or more tasks are sent to the workers with known results to quiz their output. If the output is different, then the worker is malicious; otherwise, it is trusted [11]. VIAF [11] sends multiple quizzes and ranks them or accumulates the score. The approach takes into account the overall computing behavior of each node expressed through a node weight.

Bendahmane et al. [13] proposed a technique based on the weighted t-first voting method. The approach replicates each task so that replicas are executed over multiple nodes. Then, the results are grouped according to their values. The replicated task is repeated until the result group reaches a predefined threshold (*t*). After that, workers in this group are marked as trusted. As a limitation, this technique assumes that the attacker has no knowledge about the result integrity scheme and the number of malicious workers attacking is no more than half of all available workers in the cluster. Additionally, due to the repeated computations, the approach suffers from the same high processing overhead. Moreover, it is sensitive to the choice of the threshold value (*t*).

Zhu and Lee [23] proposed a framework consisting of task replication and verification. The noncollusive workers can be detected immediately by result comparison. Therefore, they only consider collusive workers. The framework is based on defining the probability of committing cheating between colluders and/or noncolluders. If a replicated task is assigned to two collusive workers and either of them fails to pass *k* quizzes, the master will not release their results to the reducer. If a replicated task is assigned to a collusive worker and a noncollusive worker and the noncollusive worker commits a cheat, the master will not release their results to the reducer too. The master will release an incorrect result to the reducer when the two collusive map workers pass *k* quizzes and cheat in a collusive manner. The framework defines *δ* as the probability that a collusive worker will pass all of the *k* quizzes. Using *δ*, the cheat probability can be derived. Malicious workers can behave well for a long period of time to gain the trust of the master process and may attack only after that. By that time, malicious workers can pass *δ* and deceive the system. This technique still cannot guarantee the detection of all malicious mappers and reducers.

### 2.3. Replication-Based Technique

In this group of malicious worker(s) detection approaches, a task is replicated or decomposed into pieces and the pieces are replicated [24]. Whenever the task queue is not empty, the master will pick one task and send it to any two workers. After getting the two results from the two workers, the master can compare them. If the results are different, it means that at least one worker is a noncollusive worker. However, it is hard to tell which one is the noncollusive worker, but they can detect and pick the noncollusive worker later. Task replication is useless in identifying collusive workers. For detecting collusive workers, they improved the replicated task so that it is a credit-based replicated task, and they added a ` (trusted worker) to verify the intermediate results. In replication-based techniques, due to the task performed by multiple workers, system performance decreases [24, 25].

SecureMR [11] is another replication mechanism that prevents repudiation, DoS, and replay attacks. It decentralizes the integrity verification process among different distributed computing nodes which participate in the MapReduce computation. SecureMR replicates some map and reduce tasks and assigns them to different mappers and reducers; i.e., a map (or reduce) task is executed by more than one worker. SecureMR suffers from excessive processing overhead due to task replication. Moreover, this causes an overall higher latency. Additionally, it is not possible to detect collusive malicious workers.

Xiao and Xiao [15] proposed an approach that verifies every map and reduces tasks through reexecuting these tasks in a group of trusted nodes. A limitation is to have a sufficient number of trusted nodes to reperform some of the maps and reduce tasks.

### 2.4. Majority-Based Techniques

The voting-based method for identifying malicious workers sends several copies of the task to several workers [21]. The majority of voting is applied to the set of returned results to decide in favor of the result that appears most often. This approach tolerates a certain number of incorrect results in a vote. However, it does not resist a majority of colluding workers that collectively return the same incorrect result. Even though workers are randomly selected for each vote, with the possibility of massive attacks, the probability for a majority of colluders becomes significant. Ren and Tang [26] created a security module in the master node to manage the mappers based on different security levels. These levels include ordinary domain, security domain (highest level), and isolated domain (lowest level). In the beginning, mappers are in the ordinary domain. The data flow is in the ordinary domain. The execution of the task is repeated and carried out by two mappers (step 1). The verifier verifies the returned results (step 2). Upon successful verification, mappers receive a credit (step 3). Finally, the mapper's results are sent to the reducer (step 4). The mapper gains a security score when all its results are published for the reducer. Eventually, if the mapper's score reaches the security threshold, it will be promoted to the next security level. In general, tasks do not need to be replicated. Leveling out mappers has somehow contributed to enhancing security. This approach adds a number of modules in the master node and complicates the execution process. More importantly, collusive workers are not proved to be detected.

As we have explored the state of the art regarding the detection of malicious workers for MR computations, we have developed a model that guarantees the detection of colluders as well as noncolluders. In addition, we reduce the processing overhead.

## 3. Proposed Solution: MWT

In order to identify malicious workers, either collusive or noncollusive, efficiently, the proposed model is based on two facts: (1) there is no replication by quizzing with unknown solutions, and (2) the testing task shall be with small HDFS files of just one partition. This serves two objectives. First, we make sure that the mapping task will go to only one worker. Second, the resources of the cluster are not overconsumed.

### 3.1. Solution Structure

The proposed model is based on implementing a small service to be deployed in the master node called Malicious Worker Trap (MWT). It could run as a daemon program or as an integrated service with the JobTracker (see Figure 2). Our service acts as a protection layer for the cluster; it periodically performs routine checks on every worker node in the cluster in a round-robin manner. It schedules the workers one by one and repeats the checking when finished. To reduce the overhead needed for this type of checking, the service hardly requires any calculations to be performed on the master node. Instead, a list of jobs with predefined solutions is stored in the memory and used for the checking process. The frequency of the periodic check is a percentage of the workload. For example, after processing three client tasks, a checking task is sent to a worker node. Our proposed model provides a solution for a serious type of attacks when a worker behaves correctly for more than one job and then turns into a malicious worker; it periodically performs routine checks over every worker node in the whole cluster in a round-robin manner. It schedules checking the workers' nodes one by one and repeats validating them when finished in the cluster.

A list of testing tasks is defined containing the single-partition HDFS file, the program or the function, and the end result. Another list for worker nodes is required, i.e., a queue that is used to keep track of checked worker nodes. A worker node is chosen from the queue, assigned with the task and pointed to the input file. After completion by the worker node, the worker's result is compared with the stored result. Upon a match, the worker node is enqueued again for a future recheck. Otherwise, MWT sends an alert that this worker node has been infiltrated.

MWT is efficient in detecting both noncollusive and collusive malicious workers. The difficulty with detecting collusive workers is that all of them are complicit to give the wrong answer, which makes any defense technique based on the duplication of tasks ineffective. On the other hand, since our service uses a set of MapReduce jobs with predefined results, the collusion of malicious workers is detectable. Furthermore, for the case of malicious workers that act authentically for a long period of time, MWT is not only able to detect this kind of threat but also can determine the period, interval through which the cluster is endangered. This is achieved by recalling the last known right result computed by this worker, due to periodic checking. All these benefits outweigh the overhead of MWT over the workload of the cluster. MWT maintains a balance between the security and usability of the Hadoop cluster where increasing the usability of Hadoop cluster might cause risk over the system. We overcome the problem of balancing security and usability by lowering the overhead of worker validation, which can be configured as required in the system. The process of configuration helps obtain a balance between security and usability. For extra security, we use MWT service continuously, and for usability, we use MWT service only when necessary. Considering scalability, clusters can be composed on any machine in the private and/or public networks. Using machines in the public cloud hinders the security of the total system. Thus, we test each node if trusted or not by validating that the node is not malicious. When using MWT service, whether on a public or private cloud, noncollusive and collusive workers are detected, with no difference when executing the service over public cloud, private cloud, or hybrid cloud.

As stated earlier, MWT works by means of periodic checks. The frequency of these checks is a percentage of the workload, where the JobTracker is set to perform a task for the trap. This percentage is the workload occupation configuration (WOC) parameter. Based on the threats facing the system, this parameter can be altered. A list of worker nodes is required; i.e., a queue is used to log the verification process of the worker nodes.

Next, we describe how to think about the choice of WOC we build on the work in [27].

## 4. Formalization

It is clear that the available computing capabilities of different workers change over time. With high workloads, the available computing capacity goes down and new jobs start to queue up, whereas, with lower workloads, the system can accept newer jobs more frequently. So, for verification purposes, it is better to spot the time intervals with a lower workload to run the verification tasks, on the one hand. On the other hand, to reduce the risk of malicious workers, we need to detect them earlier. That is, we need to run the verification tasks more frequently. Here, the adjustment of the WOC parameter can strike a balance between the two extremes of not overloading the cluster and detecting malicious workers early enough.

In MapReduce, every map step is divided into a number of parallel tasks. Each task is assigned to a worker and is fed a partition of the input HDFS file.

Let *f*_*i*_(*t*) represent the processing speed of *i*^*t*^*h* mapper. Therefore, the total computing speed at time *t*, *p*(*t*), of the cluster using a number of *n* mappers can be represented by [27]

(1) $$\begin{array}{c} p\left(t\right)=\sum_{i=1}^{n}f_{i}\left(t\right). \end{array}$$

Let *D* represent the total amount of data for a Hadoop MapReduce job. Therefore, the computing time to process *D* can be represented through equations (2) and (3) where *a* and *b* are the endpoints of the job processing interval by the cluster:

(2) $$\begin{array}{c} \int_{a}^{b}p\left(t\right)dt\;=D, \end{array}$$

(3) $$\begin{array}{c} t=b-a. \end{array}$$

Let *w* characterize the variety of waves of mappers in the cluster to operate the whole quantity of facts *D*. In the time interval *t*, there are a wide variety of two kinds of tendencies of the processing velocity *p*(*t*). The first one is an increasing trend. We outline it as follows: from time point *t*_*a*_ to *t*_*b*_, the average processing velocity at some point of this time interval continues increasing till it gets decreased. The second one is decreasing trend. It is described as follows: from time factor *t*_*a*_ to *t*_*b*_, the average processing velocity, *P*_*ab*_, at any point during this time interval keeps reducing until it will become expanded as

(4) $$\begin{array}{c} \bar{P_{ab}}=\frac{\int_{t_{a}}^{t_{b}}p\left(t\right)\;dt}{t_{b}-t_{a}}. \end{array}$$

Thus, the algorithm selects a number for *w* that is the greatest for $\bar{P_{abt}}$:

(5) $$\begin{array}{c} p_{g}=\left\{\bar{p_{a_{1}b_{1}}},\bar{p_{a_{2}b_{2}}},\bar{p_{a_{3}b_{3}}},\ldots ,\bar{p_{a_{w}b_{w}}}\right\}. \end{array}$$

After the best values have been selected, the algorithm starts off for evolving the different two tendencies which are on the left and the proper sides of the biggest values primarily based on $\bar{P_{ab_{i}}}$ which is the wave sample in the following equation:

(6) $$\begin{array}{c} \bar{p_{a_{i-1}b_{i+1}}}=\frac{\int_{a_{i-1}}^{b_{i-1}}p\left(t\right)\text{d}t+\int_{a_{i}}^{b_{i}}p\left(t\right)\text{d}t+\int_{a_{i+1}}^{b_{i+1}}p\left(t\right)\text{d}t}{b_{i+1}-a_{i-1}}. \end{array}$$

Consequently, a number of *w* new common values $\bar{P_{a_{i-1}b_{i+1}}}$ are generated. At the same time, the wide variety of *n* tendencies decreases to the number of *n* − 2*w*. Then, in these n-2w trends, we pick out a variety of *w* best $\bar{P_{abi}}$ once more and merge the different two tendencies which are on the left and proper sides of them, till there is a range of *w* tendencies left. Therefore, the time intervals may additionally have the higher common performing capacities in the following equation:

(7) $$\begin{array}{c} T=\left\{\left(a_{1}b_{1}\right),\left(a_{2}b_{2}\right),\left(a_{3}b_{3}\right),\ldots ,\left(a_{w}b_{w}\right)\right\}. \end{array}$$

Thus, the amount of data that is executed in the time interval *t*=*b*_1_ − *a*_1_ can be transmitted to the cluster to be virtually executed. It can be predicted to be executed within a higher computing capacity interval of the cluster. The amount of data *D*1 can be represented by

(8) $$\begin{array}{c} D_{1}=\int_{a_{1}}^{b_{1}}p\left(t\right)\text{d}t. \end{array}$$

Nevertheless, because of the uncertainties and IO features of the genuine processing in the total cluster, when the quantity of facts *D*1 for the first wave is completed, the deviations of *b*1 are necessary. Hence, the expectation for the next wave is corrected. The correction method is developed as follows. In the subsequent wave, the algorithm reruns the time interval computation as defined above with modifications of values of the parameters in

(9) $$\begin{array}{c} w=w-1, \end{array}$$

(10) $$\begin{array}{c} D=D-D_{1}. \end{array}$$

Thus, with new values of *w* and *D*, a new Df can be calculated and the amount of data can be allocated to the second wave in processing. Finally, until *w* = 1, the rest of the data are allocated to the last processing wave. In a Mapper (processing unit), for processing one data block of a Hadoop MapReduce job, the total processing time could be considered through

(11) $$\begin{array}{c} T=t_{c}+t_{p}+t_{e}+t_{m}, \end{array}$$

where *t*_*c*_ represents the copying time, *t*_*p*_ represents the processor's processing time, *t*_*e*_ represents the emptying time when the buffer of the Map instance is filled up, and *t*_*m*_ represents the merging time.

## 5. Experimental Evaluation

In this section, we designed experiments to study the computation overhead of MWT. We compare the performance of MWT against Vanilla Hadoop (benchmark) and V-MR [1]. The latter has been chosen due to its recency and its superiority to the state of the art as it makes partial reexecution of some of the tasks. Our experiment solves the problems of balancing balance security and usability of the Hadoop cluster. In this experiment, we can control the use of either of the two features usability and security as desired by the system administrator. When higher security is required, then the MWT service shall send more validation tasks, i.e., before each real task. On the other hand, when the system requires more usability, the MWT service shall send validation tasks with a lower percentage between the original tasks, i.e., one-third of the time or less. Therefore, the goal is to achieve the required balance according to the system requirements.

For evaluation, and to mimic usual workloads on the Hadoop cluster, we decided to use different jobs with different complexities. These are both map-and-reduce-input heavy jobs (i.e., word count, sorting, etc.) that process enormous amounts of input data and also generate big intermediate data [27], on one side. On the other side, we will run our experiments with a different number of nodes running concurrently in the system (cluster size). This is to test the system with a different range of task loads.

### 5.1. Experiments' Setup

We performed a set of experiments analyzing the job completion time in terms of the following parameters:

- The number of nodes: 1, 10, 25, and 100
- The volume of input data: 2 GB
- The number of jobs that are executed simultaneously in the cluster: 1, 2, 3, and 4

Every node in the cluster has the same technical characteristics: 2x Intel Xeon E5-2630L v2 a 2.40 GHz, 4 GB Memory RAM, Hard disk 100 GB SATA-3, Network Intel Gigabit Ethernet.

For every experiment, we record the job completion time, fixing parameters one at a time, with permuting different numbers of workers and different data sizes. The workloads are Grep tasks, Selection tasks, and UDF aggregation tasks. This is to test the system on different volumes of data to experiment with the effect of the trap service on a system in peak time.

With the Grep task, we test the system providing different weight input user tasks (525 MB/node and 1 TB/cluster). In the Selection task, every node processes a 1 GB ranking table to retrieve the target page URLs with a user-defined threshold. In the UDF Aggregation Task, each node processes 1 GB of data. Each configuration of each task was given to MWT, Vanilla Hadoop, and V-MR. Each experiment has been repeated 5 times, and the median of completion time is recorded for the running jobs in the system.

### 5.2. Experimental Results

#### 5.2.1. Grep Task

In this type of task, we computed the execution time when each worker got 525 MB of data to process and the execution time when the whole cluster got 1 TB of data. The execution times for 525 MB per node for the different numbers of workers are reported in Figure 3. The overhead of MWT is very little in most cases. Of course, it will be higher than the vanilla MapReduce (the benchmark) but it is lower than V-MR due to the freedom from task replication and recomputation.

On the contrary, for the 1 TB of data distributed over the cluster, the execution time is plotted in Figure 4. When the load is heavy on a limited number of nodes, MWT is close to Native Hadoop while V-MR has a higher overhead, while with a large number of nodes and a highly distributed load, MWT and V-MR have comparable performance that is close to Native Hadoop.

In both scenarios, the values of the outputs are small in time intervals (in the range of 0 to 2.6 seconds in the first scenario and in the range of 4.2 to 7.5 seconds in the second scenario).

#### 5.2.2. Selection Task

The Selection task is more complex than the Grep task. In this task, in order to retrieve the target page, every node processes 1 GB ranking table. The execution time of the task for the different configurations is shown in Figure 5. The performance of MWT is close to the benchmark and faster than V-MR. The time intervals are small in the range of 2.3 and 5.3 seconds. According to this comparison between MWT, the benchmark, and V-MR results, it is clear that MWT was done at an appropriate time, taking into consideration the new service added to the JobTracker.

#### 5.2.3. UDF Aggregation Task

The UDF Aggregation Task reads the generated document files and searches for all the URLs which appeared in the contents. After that, for every unique URL, the number of unique pages will be marked to refer to a particular URL across the entire set of files.  Figure 6 shows the completion time for the job under the different configurations. It is clear that MWT overhead is very little and the overall time is close to the benchmark results, taking into consideration the complexities of the task. Still, MWT outperforms V-MR.

The experimental results show great stability of MWT outputs for the task; similar to the Grep and Search tasks, MWT results have a faster throughput than V-MR.

In conclusion, MWT result overhead is minimal compared to V-MR and close to benchmark in time. The heavier the load of the system and the higher the complexity of the load balance, the better MWT performance than V-MR.

#### 5.2.4. Discussion

Checking nodes one by one detects colluding workers to prevent them from sending false outputs to the JobTracker. For example, if there is a job requesting 20 nodes, MWT will check the 20 nodes one by one to detect the malicious workers. Commonly, a job is distributed on a number of nodes. If one of the nodes is malicious, then the job fails and the whole job has to be repeated. In MWT, the detected node task only will be repeated and not the whole work is failed and reexecuted. This is because MWT is able to check tasks per node not the whole system as a unit. If a node fails, the master can redundantly execute the same task to other nodes to avoid slow-running nodes.

In the previous approaches, trusted workers were checked before the execution of MapReduce computations, which leads to overhead, in addition to the replication overhead. With MWT, malicious workers that behave well for a long period of time to gain the trust of the master are still detectable through periodical checking of nodes one by one in a round-robin fashion.

## 6. Conclusion

Hadoop is the most common and widespread use of open-source software on a wide range of MapReduce clusters for processing huge amounts of data. There are many security issues of Hadoop MapReduce such as malicious nodes in the system. In this paper, we proposed a new model to enhance the security of Hadoop MapReduce. This model checks the workers periodically, e.g., one-third of the execution tasks of MapReduce computation, causing minimal overhead. The periodical checking model overcomes the issue of malicious workers which behave well for a long period of time to gain the trust of the master process and may attack only after that. Finally, the proposed model is able to enhance cloud security to prevent malicious and collusive workers. We evaluated the performance (i.e., overhead) on data-intensive MapReduce applications. MWT was evaluated against V-MR, a state-of-the-art malicious worker detection approach, and against Vanilla Hadoop as a benchmark. The experiments empirically prove that MWT has a lower overhead than V-MR. MWT can also be used to detect collusive and noncollusive workers in the system which improves the efficiency and effectiveness of a security module in a Hadoop MapReduce system. In future work, machine learning clustering methods will be utilized to detect the behavior of the noncollusive workers and collusive workers. Such analysis shall improve the performance of the Hadoop cluster.

## Figures and Tables

**Figure 1:** The architecture HDFS.

**Figure 2:** Structure of the MWT in the master node.

**Figure 3:** Grep task evaluation (525 MB/node).

**Figure 4:** Grep task evaluation (1 TB/cluster).

**Figure 5:** Selection task evaluation.

**Figure 6:** UDF Aggregation Task.

## Data Availability

The data used in the study can be obtained from the corresponding author upon your request.
